The article "The Intervention of Data Mining in the Allocation Efficiency of Multiple Intelligent Devices in Intelligent Pharmacy" was published in 2022. Journal: Comput Intell Neurosci.

# The Intervention of Data Mining in the Allocation Efficiency of Multiple Intelligent Devices in Intelligent Pharmacy

**DOI:** 10.1155/2022/5371575

**Published:** 2022-08-22

**Authors:** Xiaohua Li, Benren Tan, Jinkun Zheng, Xiaomei Xu, Jian Xiao, Yanlin Liu

**Affiliations:** The Affiliated Yuebei People's Hospital of Shantou University Medical College, Shaoguan 512026, Guangdong, China

## Abstract

With the wide application of artificial intelligence and big data technology in the medical field, the problems of high cost and low efficiency of traditional pharmacy management were becoming more and more obvious. Therefore, this paper proposed to use data mining technology to design and develop the dispensing process and equipment of intelligent pharmacy. Firstly, it summarized the existing data mining technology and association rule methods and expounded its application value in the related fields. Secondly, the data standard and integration platform of dispensing in intelligent pharmacy were established. Web service technology was used to design the interactive interface and call it to the intelligent device of pharmacy. Finally, an intelligent pharmacy management system based on association rule mining was constructed through the data mining of intelligent pharmacy equipment, in order to improve the intelligence and informatization of modern pharmacy management. For the emergency dispensing process of intelligent equipment failure, data mining was used to optimize the intelligent pharmacy equipment and dispensing process and change the pharmacy management from traditional prescription to patient drug treatment, so as to improve the dispensing efficiency of intelligent pharmacy equipment. Through the systematic test and analysis, the results showed that through the real-time risk prevention and control, the formula accuracy and operation speed of the intelligent dispensing machine were improved and the dispensing time was shortened. Through intelligent drug delivery, the unreasonable drug use of patients was reduced, the safety and effectiveness of clinical drug use were ensured, and the contradiction between doctors and patients was reduced. This study can not only optimize the medical experience of patients and provide patients with more high-quality and humanized pharmaceutical technical services but also provide some support for the intelligent management of modern hospitals.

## 1. Introduction

In recent years, with the rapid development of artificial intelligence and big data technology, the automation and intelligent management level of hospital pharmacies has been rising, and intelligent pharmacies have been used in some hospitals one after another. Compared with the traditional hospital pharmacy mode, the intelligent pharmacy service mode changes the traditional guarantee of drug supply into focusing on strengthening the pharmaceutical professional and technical services and participating in the dynamic management of clinical medication, so as to improve the management level of hospital pharmacy to a new level [1, 2]. In July 2018, the National Health Commission and the State Administration of Traditional Chinese Medicine issued relevant documents and encouraged qualified medical institutions to promote the construction of smart pharmacy, so as to realize the seamless connection between prescription system and pharmacy dispensing system, so as to facilitate people to take medicine in time.

The construction of intelligent pharmacy mainly involves relevant intelligent equipment, database software, and interface technology. It needs to integrate different software and hardware technologies, which has the characteristics of diversity and cross platform [3]. In the construction planning of hospital information system, the business module of the hospital is generally considered, while the overall planning of medical industry information system is less. Due to the lack of effective top-level design and standard specification requirements, there are great differences in database types and data formats involved in different information systems. At the same time, there are some problems in the construction of business information system of functional departments, such as insufficient function integration and different data interface standards, which leads to the widespread phenomenon of information island [4]. Traditional medicine management has seriously hindered the sharing of medical information and the improvement of medical service level, restricted the data sharing and resource utilization and allocation efficiency of intelligent pharmacy management information, and affected the time of taking and waiting for drugs and the quality of pharmaceutical care.

Research shows that some developed countries have effectively improved work efficiency and reduced deployment errors and labor intensity by realizing the automatic and intelligent management of pharmacies [5]. From the development trend of modern pharmaceutical industry, improving the overall application efficiency of intelligent pharmacy system and the accuracy of prescription review has become an inevitable trend of pharmacy management and development. At present, people have made a preliminary study on the intelligent efficiency of the same brand of equipment. Some people apply data mining to the market analysis, sales prediction, and intelligent drug preparation of automated pharmacies, which provides a basis for the establishment of the working mode of the automatic dispensing system of large-scale comprehensive outpatient pharmacies [6]. It is known from the existing research that the existing achievements have not conducted in-depth research on the unification of various intelligent device interfaces and data standards in the intelligent pharmacy, as well as the deployment and dispensing of various devices. Therefore, the existing intelligent drug management is still difficult to meet the needs of practical application. Therefore, this paper proposed to use data mining to study the deployment efficiency and intervention function of various intelligent devices in intelligent pharmacy, in order to provide theoretical reference for improving the modern management level and service function of intelligent pharmacy.

## 2. Related Works

With the gradual standardization of drug management under the situation of medical reform, in order to improve the capital turnover rate and reduce the cost, the hospital has adjusted the drug reserve of pharmacy accordingly. The hospital has optimized the types, quantity, and reserves of drugs, and tried to keep the balance of the use and management of drugs in stock. Through market analysis and sales forecast, some people use data mining to analyze drug sales data and inventory, and increase or decrease relevant drugs in real time, so as to maintain a dynamic balance of inventory [7, 8]. Through the given pharmacy inventory and sales data, the information is analyzed by using data mining technology, and the results are fed back to the drug warehouse, so as to effectively prevent the extrusion or shortage of drug inventory, which can not only meet the clinical needs, but also reduce the cost.

Outpatient medicine has a certain randomness. As a part of it, outpatient pharmacy should not only meet the needs of patients, but also ensure the standardized management of internal personnel. Some people use data mining technology to analyze the service information of outpatient pharmacy, and provide support for outpatient pharmacy service by evaluating the cost and risk of pharmacy. At the same time, according to the correlation degree of different links in the pharmacy service process, association rules are used to optimize relevant service matters, so as to reduce the waiting time of patients [9]. By optimizing the workflow of outpatient pharmacy, we can not only improve the allocation efficiency of drugs, but also reduce the waiting time of patients, so as to improve the service quality and level of pharmacy.

In modern intelligent pharmacy management, different types of drugs have certain differences in access efficiency. Generally, there may be some time differences when accessing the drugs in different storage locations [10]. Especially when the type and quantity of drugs change, the storage position of drugs needs to be adjusted. At the same time, the randomness of patients' demand for drugs should be fully considered in the design of pharmacy storage space. For example, patients may put forward the demand for different drugs. According to the dispensing characteristics of pharmacies, some scholars used data mining to analyze drug data and prescription information, and designed drug storage according to the batch number, distance, and relevance of drugs, and achieved certain results.

Data mining is widely used in the field of hospital pharmacy and its management [11, 12]. From the existing research results, compared with the traditional manual inference and experience, using data mining to manage the intelligent pharmacy is not only more efficient, but also more reliable. Intelligent pharmacies have high requirements for fine management and dispensing efficiency of drugs. The management of intelligent pharmacy needs the support of various intelligent devices [13]. For example, as a part of the dispensing machine, the intelligent medicine cabinet can effectively improve the efficiency and accuracy of drug dispensing only by tapping the design and functional potential of the medicine cabinet. The research shows that only by creating certain conditions for the use of intelligent medicine cabinet, can it give full play to its due effect. For example, intelligent medicine cabinet is not suitable for the storage of refrigerated drugs. Therefore, it is still difficult to obtain reliable results from drug data by using traditional data mining methods.

## 3. Data Mining Theory

### 3.1. Data Mining Method

According to the massive data provided by data warehouse and other data sources, data mining extracts the required relevant knowledge by means of mining calculation or knowledge discovery, so as to provide the basis for decision-making and analysis for relevant departments or personnel. For different research purposes, researchers' understanding of data mining may be different. Some scholars believe that the content or process of data mining and database knowledge discovery (KDD) is similar, while others believe that data mining belongs to a stage of knowledge discovery, and there are obvious differences between data mining and knowledge discovery in related connotation. This paper mainly understands data mining from the broad concept and divides it into different stages, such as data acquisition, pro-processing, data analysis, and knowledge representation.

At present, the content of data mining generally includes descriptive objects or predictive objects. Descriptive objects mainly use certain data mining algorithms to explore the correlation between data. The results explored from descriptive information need to be further verified by relevant data. Predictive data is mainly used to predict possible future events based on known phenomena, which has strong purpose. It can be seen that the descriptive information reflects the hidden law within the data, while predictive data reflects the possible results in the future.

Different from the existing data analysis methods, data mining adopts automatic statistics and analysis methods, which can not only find out the valuable information inside the data, but also predict the future development trend or change law through the obtained useful information. Data mining can analyze the correlation of massive data, which is more efficient than the traditional analysis methods. At the same time, data mining can use clustering algorithm to realize the statistical analysis of discrete data and obtain the relationship between discrete information. In addition, data mining generally processes the relevant knowledge or information under unknown conditions and obtains the results, which is completely different from the traditional data analysis methods. With the development of related technology, the analysis object of data mining is no longer limited to structured data, but extended to almost any type of data processing, such as semi-structured or unstructured data information, which provides powerful conditions for making relevant decisions in different fields.

Fayyad model and CRISP-DM model are generally adopted in the process of data mining [14, 15]. Fayyad model is divided into nine different stages: data preparation and selection, data dimensionality reduction and transformation, knowledge evaluation, and so on. The model has no specific data source and result destination in the whole process from the beginning of data processing to the final result, so its application is not strong. Different from Fayyad model, CRISP-DM model combines the specific application environment. CRISP-DM model gives a more detailed description of the data to be processed, that is, data source and selection. At the same time, it also gives application reference for the output results of the model, so as to ensure the integrity of data source, data processing, and application results. As shown in Figure 1, the basic working process of data mining is described.

In the process of data mining, the tasks to be processed mainly include data classification analysis, cluster analysis, and association analysis. Data classification mainly analyzes and processes different data to obtain the common attribute information between data, and then attribute it to different classification models [16]. Clustering mainly adopts unsupervised learning method, and uses the similarity of data to divide classes, and then classifies different data into different categories according to their attributes. Association mainly explores the internal relationship according to the attribute information between different data, so as to find the correlation between data. In practical application, parameters such as support and confidence are generally used to evaluate the correlation between different data.

### 3.2. Association Rule Mining

Association rule method is a part of data mining technology. This method is often used to deal with the internal relationship between things. It has certain stability and flexibility, and is not limited to the treatment of dependent variables. Therefore, it can provide effective support for the application of data mining in related fields [17, 18].

According to the existing research, the basic methods for association rules are as follows:

(1) If *P* and *Q* are disjoint data item sets in database *M*, that is, *P*, *Q*⊆*M*, *P*∩*Q*=Φ, then association rules can be expressed as implication in the following form:
  (1) $$\begin{array}{c} R:P⟶Q. \end{array}$$
(2) If the support of rule *Q* is expressed by *S*, *S* means that *S*% of transactions in *M* contain *P* ∪ *Q*, and the support can be expressed by *Sup*(*R*), which is as follows:
  (2) $$\begin{array}{c} \text{Sup}\left(R\right)=S\cdot M\cdot 100\%,\\ S=Sup\left(R\right),\;P\cup Q\subseteq M. \end{array}$$
(3) If the confidence of rule *Q* is represented by *T*, then *T* means that *T*% of the transactions in *M* and *N* that support *P* also support *Q*. The confidence can be expressed by Con(*R*), which is defined based on conditional probability as follows:
  (3) $$\begin{array}{c} \text{Con}\left(P⟶Q\right)=p\left(\frac{Q\subseteq N}{P\subseteq M}\right), \end{array}$$
  (4) $$\begin{array}{c} p\left(\frac{Q\subseteq N}{P\subseteq M}\right)=\frac{p\left(Q\subseteq N\cap P\subseteq N\right)}{p\left(P\subseteq N\right)}, \end{array}$$
  (5) $$\begin{array}{c} \frac{p\left(Q\subseteq N\cap P\subseteq N\right)}{p\left(P\subseteq N\right)}=\frac{\text{Sup}\left(P\cup Q\right)}{\text{Sup}\left(P\right)}. \end{array}$$

According to the above equations (3) to (5), the following relationship can be obtained:

(6) $$\begin{array}{c} \text{Con}\left(P⟶Q\right)=\frac{\text{Sup}\left(P\cup Q\right)}{\text{Sup}\left(P\right)}. \end{array}$$

If MinSup represents the minimum support and MinCon indicates the minimum confidence, when Sup(*R*) ≥ MinSup and Con(*R*) ≥ MinCon, *Q* can be considered as a strong association rule. It can be described as follows:

(7) $$\begin{array}{c} R:P\Rightarrow Q. \end{array}$$

Support is mainly used to reflect the effectiveness of association rules, while confidence is used to describe the credibility of association rules. Generally speaking, the mining of association rules should meet the minimum support threshold of user needs in order to reflect the minimum association between projects. At the same time, the confidence of mining rules should reach the lowest threshold, so that the reliability of mining rules should also reach the lowest. Therefore, the mining of association rules should reach the minimum support and minimum confidence, that is, the mining of association rules should meet the following conditions:

(8) $$\begin{array}{c} \text{Sup}\left(P\cup Q,M\right)\geq \text{MinSup},\\ \text{Con}\left(P\Rightarrow Q\right)\geq \text{MinCon.} \end{array}$$

According to the existing research, item set refers to the set of items, and *i*-item set refers to the item set containing *i* items. The sum of the number of transactions that contain the item set is called the frequency of the item set, also known as the support rate of the item set. If the item set is greater than the minimum support, it can be called a frequent item set. *D*_*i*_ represents the sum of all frequent *i*-item sets.

Mining association rules mainly include finding frequent item sets and obtaining strong association rules through frequent item sets. When searching for frequent item sets, the frequency of item sets cannot be less than the minimum support. In order to obtain strong association rules, it is necessary to ensure that the rules are greater than the minimum support and minimum confidence.

Association rule mining methods can be classified from different angles. Firstly, in terms of the types of variables handled by association rules, association rule mining methods can be divided into Boolean and numerical types [19]. Boolean association rules mainly deal with discrete objects. This method only considers the existence of data items without knowing the number of data items. Numerical association rules mainly deal with the relationship between data items. The data item set processed by this method contains at least one data item belonging to numerical type. Secondly, from the data abstraction level processed by association rules, association rule mining methods can be divided into single-level association mining and multi-level association mining. The data items processed by the single-level association mining method belong to the same level, while the data items processed by the multi-level association mining method may belong to different levels. In addition, according to the data dimension processed by association rules, association rule mining methods can be divided into single-dimensional association mining and multi-dimensional association mining. If the attribute of the processed data item is single, the association rule mining is single-dimensional association mining. If the attribute of the processed data item is multiple, the association rule mining is multi-dimensional association mining. The object processed by the single-dimensional association mining method is the relationship between single attributes, while the object processed by the multi-dimensional association mining method is the relationship between multiple attributes.

### 3.3. Association Rule Algorithm

Apriori algorithm can be used to get the required frequent item sets and obtain the corresponding association rules. Apriori algorithm mainly finds all frequent item sets through two different stages. Apriori algorithm forms the preliminary item set with the length of *i*+1 from the frequent item set with the length of *i* through the layer-by-layer iterative method, and then forms the frequent item set with the length of *i*+1, so as to obtain the corresponding association rules [20].

After setting the minimum support, start running the Apriori algorithm. First, calculate the support of each item one by one through scanning to form a frequent 1-item set, and then traverse *i* times until the obtained frequent item set is empty, and then stop the algorithm. The running process of Apriori algorithm is shown in Figure 2.

Apriori algorithm needs to scan the database many times in the process of data mining, which brings a large workload to the input and output of data. Moreover, Apriori algorithm may produce a large number of pre-selected item sets in the running process, which increases the running time and memory overhead of the algorithm to a certain extent. Therefore, FP-tree algorithm can be used, which can effectively obtain the association rules by generating frequent item sets [21, 22].

In order to improve the efficiency of obtaining the association rules, some people improve FP-tree algorithm and propose FP-growth algorithm. When using this algorithm, firstly, the database is scanned once, and the generated frequent item sets are added to the frequent pattern tree. Then, the association information between item sets remains unchanged. Then, the generated FP-growth is divided into different condition trees, and each condition tree corresponds to a frequent item set. Finally, the condition trees are mined in turn. FP-growth algorithm can be effectively applied to different rules, and it is better than the other algorithms in efficiency.

## 4. Deployment of Multiple Intelligent Devices in Intelligent Pharmacy

### 4.1. Construction of the Data Integration Platform for the Intelligent Pharmacy System

Web service is an Internet-based development model proposed by Microsoft [23]. It provides services for other applications through web communication protocol and open standards of information format (HTTP, XML, and soap). The integrated platform involves software suppliers such as his system (Beijing Donghua, cache database, and software architecture B/S), Tangshan automatic medicine dispenser system (Japan, SQL Server database, and software architecture C/S), medicine taking and reporting machine system (Great Wall, MySQL database, and software architecture C/S), Weilehitz whole box dispensing consis system (Shanghai, SQL database, software architecture is dbo), and Shenzhen weisi'an drug intelligent management system. The system interface technologies include WebService, XML, WebService + XML.

After data mining the information stored by various intelligent devices, the format and interactive content of pharmacy data information can be further unified, and the corresponding interface program can be developed. Collect the interface documents of all intelligent devices and establish a unified pharmacy dispensing database. The main data tables are as follows:

1. *Basic Data Sheet of Drug Information*. This table mainly includes drug code, alias, trade name, English name, category, dosage form, specification, minimum specification, packaging unit, large packaging unit, packaging conversion factor, dose unit, minimum unit dose, dose conversion factor, drug price, manufacturer, manufacturer code, approval number/registration certificate number, storage conditions, storage type, and stop sign.
2. *Pharmacy Drug Storage Location Data Sheet*. This table mainly includes drug number, storage location information, drug batch, drug batch number, production date, expiration date, and storage location inventory quantity.
3. *Hospital Department Basic Data Sheet.* This table mainly includes department number, department name, and department category.
4. *Pharmacist Basic Information Data Sheet*. This table mainly includes pharmacist number, pharmacist job number, department number, pharmacist name, professional title, and job category.
5. *Prescription Information Data Sheet*. This table mainly includes prescription time, prescription number, patient name, medical card number, invoice number, patient type, patient birth date, patient gender, patient identity, medical insurance type, prescription attribute, prescription type, diagnostic information, prescription remarks, number of doses, expenses, paid in expenses, billing department number, billing department name, prescribing doctor, dispensing priority, drug name, drug specification, manufacturer number and manufacturer name, drug packaging specification, drug packaging unit, drug dose, dose unit, drug usage, drug dosage, supplementary usage, prescription details, and remarks.
6. *Prescription Window Information and Screen Call Information Data Sheet*. This table mainly includes dispensing window, dispensing time, dispensing man number, dispensing person's name, call number display information, drug return time, quantity, drug return person's name, and work number and other information.

In order to meet the various needs of pharmacies, intelligent pharmacy equipment and its control system can be used to improve the prescription allocation efficiency and information management level of modern hospitals. The intelligent pharmacy uses semi-automatic equipment to receive the electronic prescription provided by the hospital management system. Through data mining and information association processing, it compares the drug information stored in the upper computer, sends relevant instructions to the lower computer through the data bus, allocates the drugs required by the patients to the drug outlet, reminds relevant personnel to extract the corresponding drugs, and then transmits them to the patients from the drug distribution window after verification.

The intelligent pharmacy control system is mainly composed of upper computer control and lower computer control. Its control system and distribution are shown in Figure 3.

In the intelligent pharmacy control system, the upper computer system mainly receives and processes the prescription information from the hospital by using the data mining method, obtains the drug distribution in the dispensing prescription by associating the data, and then sends instructions to the lower computer system. Then, allocate the corresponding bin to the medicine outlet for relevant personnel to take medicine for dispensing, and receive the feedback message from the lower computer at the same time. When the drug treatment is finished, send the prescription to the window, and return the prescription to the patient after the relevant personnel check the dispensing prescription. The lower computer system mainly receives the instructions from the upper computer system and processes them through data mining. Then, send the instruction to the corresponding intelligent device, transfer the instruction to the drug outlet through the corresponding bin of the device, and display the corresponding instruction and drug information on the man–machine interface board for the staff to take the medicine. When the above operations are completed, the results are transmitted to the upper computer system to feed back relevant information.

### 4.2. Intelligent Pharmacy Management System Based on Association Rule Mining

Association rule mining for medicine is mainly based on the prescription drug information provided by the hospital database to mine the information hidden between drugs with certain association. Because the hospital medical database stores a large amount of information occurring in the medical process, including clinical medical diagnosis information and medical management information, the medical data information has a wide range of sources and a large scale. Medical data information usually has certain characteristics. Medical data usually show some heterogeneity and complexity, and medical academic language is relatively rich, which brings some difficulties to the processing of medical information by data mining. Medical data has certain privacy, that is, the privacy of patients. In the process of data mining, we should not only protect the privacy of patients, but also ensure the security of relevant data. Medical data has certain diversity, that is, the establishment of medical database is based on medical experimental observation, doctor diagnosis, and communication between doctors and patients. Therefore, medical data have various forms, which is also the characteristic of medical data different from other types of data information. Medical data has certain relevance, that is, the data in cases may be related to each other. For example, there is often correlation between symptoms, therapies, prescriptions, and drugs, which can be explored by association rule mining. Medical data has certain repeatability, that is, the case data stored in the medical database will inevitably have some duplicate information. Association rule mining method can be used to find the hidden rules in the data. It can be seen that although a large number of medical data are diverse and complex intertwined, on the basis of data pro-processing, association rules can be used to mine the internal laws of medical data.

Considering that the purposes of data mining may be different in practical application fields, the process of data mining is related to specific application fields. For medical data mining, mainly according to the medical information resources stored in the hospital database, the data mining algorithm is used to mine the knowledge with certain correlation between the data. The specific mining process of medical data is as follows:

First of all, make relevant preparations and clarify the main objectives and work steps of medical data mining. On the basis of mastering the characteristics of medical data, pro-process the information stored in medical database with standardization and structure, so as to provide effective guarantee for the mining of association rules. Secondly, according to the goal of medical data mining, appropriate data mining algorithms are used to obtain the required information, and the mining results are analyzed and evaluated. Finally, test the results, decide whether to further mine the medical data according to the feedback results, and apply the final data mining results to the actual system.

As shown in Figure 4, it reflects the framework of intelligent pharmacy management system based on association rule mining.

### 4.3. Optimization of the Intelligent Pharmacy Management System

Based on the constructed data integration platform and intelligent pharmacy, the original dispensing process of pharmacy can be further optimized, and the integrated platform and unified data standard can be developed. At the same time, the dispensing process of outpatient prescriptions and emergency prescriptions can be improved by using the standard interface provided by intelligent devices, as shown in Figures 5 and 6.

Considering that various devices in the intelligent pharmacy may fail during use, the emergency dispensing process in case of failure of intelligent devices in the pharmacy is optimized through the construction of data integration platform.

## 5. System Test and Result Analysis

### 5.1. System Integration

In 2018, the outpatient pharmacy of our hospital carried out the transformation and construction of intelligent pharmacy, and introduced the first fully automatic integrated dispensing machine, intelligent medicine rack, transportation track, and other intelligent and automatic advanced equipment of pharmacy in Japan. The his system is connected with the pharmacist workstation, which realizes the preliminary intellectualization and automation of drug dispensing in the hospital, and changes the existing mode of manual dispensing and distribution of drugs in the hospital pharmacy. In 2021, weilehitz (Shanghai) was introduced to integrate intelligent equipment such as dispensing machine, and an integrated platform was built by using web service technology to integrate all kinds of servers, high-performance processors, and medical databases through the development and management environment system. According to the prescription data characteristics of various intelligent devices in intelligent pharmacy, data mining technology is used to analyze the relevant information, so as to improve the intelligent degree, dispensing efficiency, dispensing speed, and quality of pharmacy.

### 5.2. Result Analysis

#### 5.2.1. Comparative Analysis of Equipment Faults

The equipment failures and errors of the dispensing machine from July to September 2020 were statistically analyzed. The main problems occurred in the whole machine drug receiving basket, drug delivery, drug delivery receiving basket, transmission process, drug lifting, machine restart, drug filling, and other links. In view of various problems, the replacement or transformation and upgrading of relevant equipment were carried out, and the faults and errors of the optimized intelligent pharmacy equipment were statistically analyzed from July to September 2021. The results showed that the failure rate of the system was reduced by 45.27% on average, which effectively improved the operation stability of intelligent pharmacy. The comparison results of faults and errors before and after optimization of intelligent pharmacy equipment are shown in Table 1.

#### 5.2.2. Analysis of Allocation Efficiency

From July to September 2020, the medical data sent by HIS system received by the dispenser every day were mined and analyzed, and the difference between the prescription payment time of patients in the outpatient department and the dispensing processing time of the dispenser was compared. As shown in Figure 7, it was the average waiting time of patients before building the data platform. Through data mining and association rule processing, the main reasons for the delay of dispensing machine were obtained. These factors mainly included the slow dispensing speed of the dispenser itself, the lack of drugs, the blockage of the dispensing basket due to the failure of the dispensing personnel to take drugs in time at the peak, and the blockage of the transportation of the medicine basket due to the failure of the dispensing personnel to take drugs in time. In addition, the deployment delay may also be caused by the networking delay of drug dispensers, drug errors, basket string, etc.

Aiming at the problem of dispensing delay of dispensing machine, this paper used data mining to analyze the prescription data of various intelligent devices in intelligent pharmacy, adopts data integration management, and optimized the dispensing machine and other intelligent devices in pharmacy. Then, the medical data were mined and analyzed from July to September 2021, and the waiting time of patients was compared. As shown in Figure 8, it was the average waiting time of patients after building the data platform. According to the comparison results of the average waiting time of patients before and after the construction of the data platform, it was known that the intelligent pharmacy after the construction of the data platform can significantly improve the dispensing efficiency, dispensing speed, and quality.

Through the construction of data integration platform and prescription data mining, the use of various intelligent devices in the pharmacy had been optimized, the dispensing efficiency of the pharmacy had been improved, and the waiting time of patients in peak hours had been shortened.

## 6. Conclusion

This paper studies the design and development of intelligent pharmacy, and establishes the dispensing data standard and integration platform of intelligent pharmacy. Web service technology is used to design the interactive interface, which can be called by various intelligent devices. It is also used to standardize the emergency dispensing process of various intelligent equipment failures, optimize the intelligent pharmacy equipment and dispensing process by using data mining, and improve the dispensing efficiency of intelligent pharmacy equipment. Through the data mining of intelligent pharmacy equipment, the intellectualization and informatization of modern pharmacy management are improved. Change the pharmacy management from traditional prescription based to patient-centered drug treatment. Through real-time risk prevention and control, the formula accuracy and operation speed of the intelligent dispensing machine are improved, and the dispensing time is shortened. Through intelligent drug delivery, the unreasonable drug use of patients is reduced, the safety and effectiveness of clinical drug use are ensured, and the contradiction between doctors and patients is reduced. The research results obtained in this paper can not only reflect the professional technical value of pharmacists and change the pharmaceutical care mode, but also optimize the medical experience of patients, so as to provide patients with more high-quality and humanized pharmaceutical technical services. This study can provide some reference for modern hospital intelligent management and its economic and social benefits.

## Figures and Tables

**Figure 1:** The basic working process of data mining.

**Figure 2:** The running process of apriori algorithm.

**Figure 3:** Structure and distribution diagram of the intelligent pharmacy control system.

**Figure 4:** The framework of intelligent pharmacy management system based on association rule mining.

**Figure 5:** Outpatient prescription dispensing process after system optimization.

**Figure 6:** Emergency prescription dispensing process after system optimization.

**Figure 7:** Average waiting time of patients before building the data platform.

**Figure 8:** Average waiting time of patients after building the data platform.

**Table 1:** Comparison results of faults and errors before and after optimization of intelligent pharmacy equipment.

Fault type	2020			2021		
	July	August	September	July	August	September
Machine drug receiving basket	135	58	39	107	32	12
Drug delivery	78	52	43	38	26	5
Drug delivery receiving basket	97	36	41	63	18	14
Transmission process	59	57	38	25	23	9
Drug lifting	76	47	44	39	15	13
Machine restart	73	56	47	42	23	7
Drug filling	54	42	35	21	14	8
Other links	42	39	47	14	12	6

## Data Availability

The labeled data set used to support the findings of this study is available from the corresponding author upon request.
